# Association between the salinity level with miscarriage and unintended pregnancy in Bangladesh: Impact of salinity level on miscarriage and unintended pregnancy in Bangladesh

**DOI:** 10.1016/j.heliyon.2023.e23858

**Published:** 2023-12-18

**Authors:** Sorif Hossain, Md Abid Hasan, Mohammad Omar Faruk, Muhammad Abdus Salam

**Affiliations:** a Department of Statistics, Noakhali Science and Technology University, Noakhali- 3814, Bangladesh; b Department of Oceanography, Noakhali Science and Technology University, Noakhali-3814, Bangladesh; c Department of Management Information Systems, Noakhali Science and Technology University, Noakhali-3814, Bangladesh

**Keywords:** Salinity, Miscarriage, Unintended pregnancy, Coastal areas, Bangladesh

## Abstract

Miscarriage is a significant public health concern worldwide, particularly in developing nations like Bangladesh. Moreover, people in coastal areas are more affected by miscarriage as compared to other areas. Increasing sea levels and salinity is the main reason for this discrepancy. This study aimed to investigate the association between different salinity levels (S1, S2, S3, S4, and S5) and miscarriage and unintended pregnancy. The outcome variables are pregnancy-related outcomes (miscarriage, unintended pregnancy), and the independent variables are different salinity levels. A frequency table and correlation analysis were done to find the descriptive scenarios of miscarriage, unintended pregnancy, and salinity levels. We found 621 miscarriage patients and 2271 unintended pregnant patients in our study. Furthermore, the Poisson regression model was used to observe the incidence of miscarriage and unintended pregnancy for different salinity levels. A higher amount of miscarriage and unintended pregnancy rate was found in Dhaka and Khulna, while these rates were lower in Barisal and Chittagong. However, the salinity levels were highest in Barisal and Khulna. Both miscarriage and unintended pregnancy are highly and negatively correlated with salinity levels. The Poisson regression model shows that the salinity levels s1-s5 are strongly associated with miscarriage. Lower and moderate levels of salinity are strongly associated with miscarriage than higher levels of salinity. Again, the average number of miscarriages decreases with the salinity levels. Likewise, unintended pregnancy was also negatively associated with salinity levels. However, it only reported a significant association with lower and moderate salinity levels, and higher salinity levels did not affect unintended pregnancy. Taking initiatives for raising awareness from government and non-government organizations, setting up deep tube water pumps extensively, and properly treating coastal areas women during pregnancy would be the ideal next step to reduce the miscarriage and unintended pregnancy rate in coastal zones in Bangladesh.

## 1 Introduction

Miscarriage is frequently subject to misinterpretation among a significant number of women, men, and medical professionals, resulting in the prevalence of misconceptions around this phenomenon [1,2]. The term "miscarriage" often refers to the termination of a pregnancy within the uterus before the point of fetal viability. However, some difficulties are associated with accurately diagnosing pregnancy and establishing clear criteria for determining if a pregnancy is indeed intrauterine and whether the fetus has reached a stage of viability [3]. The duration of conception or fetal weight can determine the survivability threshold. The gestational limits for viability vary across different geographical regions, often falling within an interval of 20–28 weeks of conception. According to the World Health Organization (WHO), miscarriage is characterized as the involuntary termination of a pregnancy, resulting in the evacuation or extraction of a fetus (sometimes referred to as an embryo) with a weight below 500 g, which is roughly comparable to a gestational age of around 22 weeks [4,5]. An unexpected pregnancy, on the other hand, refers to a pregnancy that is characterized by either being undesired, implying that it occurs when individuals do not wish for any or any further children, or being mistimed, indicating that the pregnancy occurs sooner than anticipated [6]. The notion of unwanted pregnancy is crucial in comprehending individuals' fecundity and the prevalence of unmet contraceptive needs, also referred to as birth control. The majority of unwanted births arise due to either the lack of utilization of contraception or the inconsistent or incorrect usage thereof [7].

Bangladesh is a low-lying deltaic nation where the contamination by saltwater from the Bay of Bengal threatens natural drinking water supplies, including rivers and groundwater [8]. Although salt (NaCl) is an essential mineral that has a considerable impact on human health and diseases, the recommended daily intake of salt is below 5 g (2000 mg of sodium) for adults and lower for children [9,10]. Excessive salt consumption is a key contributor to hypertension and associated illnesses, such as cardiovascular disease and stroke [11,12]. Preeclampsia and miscarriage are the most prevalent complications of pregnancy. The two categories of miscarriage are sporadic and recurrent. Around 50% of the women suffer from sporadic miscarriage, while 01% undergo the recurrent symptoms [13]. Miscarriage has multiple causes; among them, inflammatory and immune system problems are major contributors [13]. Preeclampsia results in hypertension, proteinuria, and renal issues. About three to five percent of women have preeclampsia. Prenatal fatalities, maternal morbidity, and maternal deaths are all significantly attributed to preeclampsia [14]. Most recent studies expressed salts' role in miscarriage and Preeclampsia. Studies have also shown that salt is crucial in exacerbating inflammatory procedures and increasing autoimmunity [15]. Numerous research has also clarified how the inflammatory process contributes to the development of preeclampsia and miscarriage [16].

The effects of climate change are already seen in Bangladesh, making it one of the world's most vulnerable nations. Being a riverine country with a coastal region incorporating a portion of the flat Ganges delta, it flows a significant amount of water into the Bay of Bengal. The rising sea level and salinity intrusion are currently threatening approximately 30% of the arable lands of coastal Bangladesh, where direct inundation, tidal flooding, and the transportation of salt-affected surface and groundwater are known to be influencing groundwater salinity [17]. The saline water of the Bay of Bengal endangers the primary drinking water resources of coastal Bangladesh, such as rivers, lakes, and tube wells. More than 20 million coastal inhabitants are affected by the fluctuating salinity of drinking water from these distinct natural reservoirs. The Integrated Regional Information Networks (2007) reports that since 1948, river salinity in the southern regions of Bangladesh has increased by 45 percent. Recent research in the different coastal areas revealed that the accumulated lands were generally high to severely salty (ranging from 1.35 to 4.70 dS/m) at 45–60 cm depth [18]. Multiple studies have also discovered evidence of salinity across several coastal areas [[19], [20], [21]]. We anticipate a greater miscarriage incidence in the coastal belt of these areas, which has been affected by salinity intrusion.

Hypertension from high salt consumption via drinking water in coastal regions could be dangerous during pregnancy. If hypertension is not treated, it may result in serious pregnancy-related issues, leading to late pregnancy failure or even miscarriage. This study aims to examine the effects of groundwater salinity on the occurrences of miscarriage. A 2011 study [22] identified a relationship between excessive salt consumption and the emergence of gestational hypertension and preeclampsia. However, the association between excessive exposure to salt and miscarriages is yet to be investigated. Thus, the primary objective of this study is to explore the impacts of salinity levels on the incidence of miscarriage within the coastal regions of Bangladesh. Moreover, this research aims to analyze the relationship between different salinity levels (S1, S2, S3, S4, and S5) with miscarriage and unintended pregnancy.

## 2 Methodology

### 2.1 Sampling design

This study selected districts as the primary sampling unit (PSU) and Upazilla as the secondary sampling unit (SSU). The salinity measurements S1–S5 (Lower-higher saline area) were estimated for 2011 for each Upazilla. The loss of birth information was collected from DHS datasets for the same year and Upazillas [23]. The DHS program conducted a cluster survey of each district. Each district was considered a PSU, and Upazilas were considered an SSU. This study extracted information on miscarriage and unintended pregnancy of married women aged between 15 and 49 from the DHS dataset.

### 2.2 Data collection

This study collected secondary observational data due to the lack of a laboratory to test the salinity at the soil level. The salinity information for 2011 and the specific geographical location (especially coastal areas) were collected from the soil science department and the head of the salinity center in Khulna. The salinity data was collected for the Barisal, Chattogram, Dhaka, and Khulna divisions. The miscarriage and unintended pregnancy information for these specific districts (Barisal, Chattogram, Dhaka, and Khulna) was collected from Bangladesh Demographic and Health Survey 2011 (BDHS) data found at the Bangladesh Bureau of Statistics (BBS) [23]. This investigation found 621 miscarriage patients and 2271 unintended pregnant patients in the selected areas. The BDHS 2011 data was used in this investigation because we only have salinity information in 2011 and observed the association for the particular year.

### 2.3 Outcome variables

The study outcome was miscarriages, defined as loss of pregnancy before or equal to 20 weeks, [24]. We also considered unintended pregnancy as another outcome variable. Both of our outcome variables were continuous variables which count the total number of miscarriage and unintended pregnancy over the division. An unexpected pregnancy is unwanted, or no further children are desired [25].

### 2.4 Independent variables

Salinity levels s1 (2–4 ds/m), s2 (4.1–8.0 ds/m), s3 (8.1–12.0 ds/m), s4 (12.1–16 ds/m), and s5 (>16.1 ds/m) were considered as explanatory variables, which determine low saline area (s1) to high saline area (s5).

### 2.5 Statistical analysis

This study used crosstabs to see the different scenarios of miscarriage and unintended pregnancy rates with salinity levels. Correlation analysis was performed to find if there is any linear association between miscarriage and salinity levels. Moreover, the Poisson regression models were used to find the association between miscarriage and unintended pregnancy with salinity levels. R (4.4.0) and STATA (16.0) software were used to conduct the analysis.

## 3 Results

The majority of miscarriages and unintended pregnancies occurred in Dhaka (211, 650) and Khulna (156, 599). However, the salinity level was higher in Barisal as compared to other divisions. The salinity level was lowest in Dhaka, and this division was not associated with higher salinity levels as s4 and s5 are zero (Table 1). As shown in Fig. 1, the miscarriage and unintended pregnancy rates varied in different regions. The miscarriage and unintended pregnancy rates were higher in Dhaka and lower in Barisal. However, Dhaka regions reported low salinity levels, whereas the Khulna region found high salinity levels (Fig. 2).

**Table 1:** Total number of miscarriages and salinity levels in Bangladesh.

Division	Miscarriage	Unintended pregnancy	s1 (2–4 ds/m)	s2(4.1–8.0 ds/m)	s3(8.1–12.0 ds/m)	s4 (12.1–16 ds/m)	s5 (>16.1 ds/m)
Barisal	104	445	166510	112540	52530	42520	24080
Chittagong	150	577	47090	48800	41940	34250	9450
Dhaka	211	650	4380	950	60	0	0
Khulna	156	599	107840	108800	94650	85210	68390

**Fig. 1:** Spatial mapping of miscarriage and unintended pregnancy in different divisions.

**Fig. 2:** Spatial mapping of salinity levels in different divisions.

Miscarriage and unintended pregnancy were highly and negatively correlated with salinity levels. However, this correlation was lower with a higher level of salinity. For example, the correlation between miscarriage and s1 was −0.90, whereas this correlation was −0.30 with s5. Similarly, the correlation of unintended pregnancy with s1 was 9 times higher than s5 (Table 2).

**Table 2:** Correlation between miscarriage and unintended pregnancy and salinity levels.

Salinity Level	s1	s2	s3	s4	s5
Miscarriage	−0.90	−0.84	−0.55	−0.50	−0.30
Unintended pregnancy	−0.87	−0.70	−0.30	−0.24	−0.09

The Poisson regression model showed that the salinity levels s1-s5 were strongly associated with miscarriage (Table 3). Lower (S1–S2) and moderate salinity (S3–S4) levels were strongly associated with higher salinity levels. The mean number of miscarriages decreased with the salinity levels. The lower salinity levels, such as S1 and S2, were intensely associated (p-value<0.001) with miscarriage and unintended pregnancy as compared to moderate (p-value<0.05) and higher salinity levels (p-value<0.10). The mean number of miscarriages decreased by −3.72e-06 units with lower salinity levels, whereas it decreased by −2.98e-06 units with higher salinity levels. Moreover, lower salinity levels showed a more significant influence on miscarriage than higher salinity levels.

**Table 3:** Poisson regression model estimate for both miscarriage and unintended pregnancy.

		Estimate (95%CI)	
		Miscarriage	Unintended Pregnancy
	S1	−3.72e-06*** (−5.05e-06, -2.40e-06)	−1.93e-06*** (−2.61e-06, -1.25e-06)
**Salinity levels**	S2	−4.34e-06*** (−6.01e-06, -2.67e-06)	−2.01e-06*** (−2.89e-06, -1.14e-06)
	S3	−4.05e-06** (−6.40e-06, -1.70e-06)	−1.20e-06* (−2.43e-06, 1.80e-08)
	S4	−4.08e-06** (−6.71e-06, -1.44e-06)	−1.08e-06 (−2.44e-06, 2.85e-07)
	S5	−2.98e-06* (−6.09e-06, 1.19e-07)	−4.71e-07 (−2.05e-06, 1.11e-06)

p < 0.001***, 0.001<p < 0.05 **, 0.05<p < 0.10*.

Likewise, unintended pregnancy was also negatively associated with salinity levels. However, it only reported a significant association with a lower (S1–S2) and moderate salinity (S3–S4) level. Higher salinity levels (estimate = -4.71e-07, 95 % CI = -2.05e-06-1.11e-06) did not affect unintended pregnancy (Table 3).

## 4 Discussion

The rising sea levels and associated repercussions have become progressively more apparent in recent years. Based on the findings of environmental experts, it has been observed that there is a direct relationship between the rise in sea level and the decrease in atmospheric pressure, with a rate of 10 mm of sea level rise for every millibar decrease in atmospheric pressure [26]. Bangladesh is a nation that faces significant challenges due to the adverse impacts of increasing sea levels associated with climate change, and these challenges have led to the emergence of elevated salinity levels along the coastal regions of the country [27]. Moreover, a notable correlation exists between elevated salt levels and many health conditions, including but not limited to miscarriage, unplanned pregnancy, and stillbirth.

The Sustainable Development Goals (SDGs), often mentioned as the Global Goals, were formally advocated by the United Nations in 2015, which function as a thoroughgoing and inclusive agenda, advocating for coordinated attempts to eliminate poverty, protect the environment, and advance peace and prosperity for all by 2030 [28]. The scopes of this investigation align closely with goal three, which pertains to promoting good health, and goal six, which refers to ensuring clean water. Despite Bangladesh's notable achievements in areas such as poverty alleviation, gender parity, access to electricity, sanitation, yearly GDP growth, and public health, a considerable proportion of pregnancies in the country continue to result in miscarriages [29]. Based on a recent study conducted by the International Centre for Diarrhoeal Disease Research, Bangladesh (ICDDR, B), it has been determined that in the region of Chakaria, the rate of miscarriages during pregnancy amounts to 11 %. The researchers arrived at the additional conclusion that the occurrence of miscarriages is more probable in proximity to coastal areas, which can be attributed to the higher salt content present in the drinking water [30]. According to the guidelines set out by the World Health Organization (WHO), limiting daily salt intake to a maximum of 5 g is advised. Multiple research investigations have attempted to determine the mean daily salt consumption of individuals residing in Bangladesh, with none reporting a number lower than 5 g [31]. While it is possible that other variables may contribute to miscarriage, our study has established a clear and direct correlation between miscarriage and salinity.

“In an effort to maintain consistency with the data clustering methodology employed in the Bangladesh Demographic and Health Survey, we endeavored to arrange the salinity data in a comparable manner. Despite the absence of in-situ measurements for salinity, we obtained salinity data for the designated year and geographic location from two reputable data repositories. One notable strength of this research is its comprehensive coverage, encompassing a significant portion of the country, including the divisions of Barisal, Chattogram, Dhaka, and Khulna, which collectively account for over fifty percent of the nation's territory. Furthermore, the salinity levels were categorized into five unique classes, facilitating our comprehension of the impacts of varying salinity levels on the occurrence of miscarriages and unwanted pregnancies. To gain a comprehensive understanding of various instances of miscarriage and unwanted pregnancy in relation to salinity, we employed crosstabulation analysis to compare and contrast the findings. The correlation analysis and Poisson regression models were significant for comprehending the relationship between miscarriage and unplanned pregnancy concerning salinity levels. The findings of our study indicate a significant inverse relationship between salinity levels and the occurrence of both miscarriages and unwanted pregnancies, which was also observed to decrease with rising salinity levels. Although Barisal and Khulna are the two divisions predominantly affected by salinities, Dhaka was recorded to be the division that possesses the maximum number of miscarriages and unintended pregnancies.

### 4.1 Strength

This study's main strength is the new study for Bangladesh perspectives. No study has been conducted yet to show the association between salinity levels with miscarriage and unintended pregnancy. Moreover, this study used spatial mapping to understand the salinity levels and miscarriage and unintended pregnancy rates over the regions. Furthermore, this study observes the miscarriage and unintended pregnancy rates for lower to upper salinity levels, which is a new insight in this study.

### 4.2 Limitations

According to the previous literature review, the miscarriage and unintended pregnancy rates were increasing with salinity levels, and it was higher in coastal regions than in their counterparts. However, these results contradict our present study. We found the highest number of unintended pregnancies and miscarriage rates with lower salinity levels in some cases. This might be the reason for lower health facilities and consciousness in those areas [32]. We only considered salinity levels as an explanatory variable for predicting miscarriage and unintended pregnancy rates. However, many variables can impact the miscarriage rate, which we didn't consider in our study. In our study, we also didn't consider sociodemographic and socioeconomic and health-related variables number of infants ever born, age of the mother at the time of interviewing, mother's employment status, her marital status, mother's body mass index (BMI), level of education of her parent, mother's age at the time of the index childbirth, her desire for pregnancy, and mother's access to media (television, radio or newspaper), which also have an intense impact on miscarriage and unexpected pregnancy rate [33]. Furthermore, we collected data from only some regions in each district, which was insufficient to reveal the real causes of salinity levels on health impacts. Miscarriage data and unintended pregnancy information were only available at the division levels. That is why we couldn't capture the real association with them. Another limitation was we used only 4 observations to estimate the parameters from poisson regression model. Although we had 102 Upazilas information for salinity levels, unfortunately we only obtained division levels data in the BDHS 2011 data sets. Our observations number was also limited and need to explore more by using more sample numbers. Since our observations number was small, we can't make stable conclusions regarding this study and need to explore this study further.

## 5 Conclusions

Efforts and resources are evidently essential for initiatives aimed at addressing miscarriages and unintended pregnancies, with particular focus needed on coastal regions and women's health. While formal studies assessing the direct link between these issues are lacking, it is undeniable that the support provided by these programs contributes significantly to improving access to clean water. Consequently, this support plays a crucial role in reducing unintended pregnancies and lowering the miscarriage rate. From this study, it can be inferred that salt levels impact pregnancy outcomes, with a more significant effect observed in Bangladesh coastal areas. To reduce the rate of miscarriages and unintended pregnancies in Bangladesh's coastal areas, the ideal next step would be for government and non-government organizations to increase public awareness. Many deep-tube water pumps would need to be installed, rainwater harvesting strategies should be promoted, and pregnant women living in coastal areas would need proper care. The increasing salt levels have prompted a heightened awareness and a surge of interest in the effects of climate change on water supplies. There is a growing advocacy for implementing adaptation techniques to enhance coping mechanisms and mitigate community vulnerabilities. Further investigation is necessary to thoroughly comprehend the impacts of salinity on pregnant individuals and enhance the administration of surface and groundwater reservoirs.

## 6 Suggestions for future research

Extensive research should be accomplished by collecting water salinity levels and birth-related information from all coastal zones in Bangladesh. Gathering data from only some places will mask the real effect of salinity levels on pregnancy problems, which we already mentioned in our study. Further research can be conducted by collecting miscarriage and unintended pregnancy information in the Upazilas levels to get the precise estimate of the parameter.

## Ethical statement

The authors did not personally collect data for this study. This study was conducted using secondary data sets.

## Funding

This research received funding from Research Cell, Noakhali Science and Technology University, Bangladesh.

## Data availability statement

Data will be made available upon request.

## CRediT authorship contribution statement

**Sorif Hossain:** Writing - review & editing, Writing - original draft, Visualization, Validation, Supervision, Software, Resources, Project administration, Methodology, Investigation, Funding acquisition, Formal analysis, Data curation, Conceptualization. **Md Abid Hasan:** Writing - review & editing, Writing - original draft, Visualization, Validation, Supervision, Methodology, Investigation, Formal analysis, Conceptualization. **Mohammad Omar Faruk:** Writing - review & editing, Writing - original draft, Visualization, Validation, Supervision, Resources, Project administration, Investigation. **Muhammad Abdus Salam:** Writing - review & editing, Writing - original draft, Project administration.

## Declaration of competing interest

The authors declare that they have no known competing financial interests or personal relationships that could have appeared to influence the work reported in this paper.
